RETRACTED

# Modern Virtual Fencing Application: Monitoring and Controlling Behavior of Goats Using GPS Collars and Warning Signals

**DOI:** 10.3390/s19071598

**Published:** 2019-04-02

**Authors:** Azamjon Muminov, Daeyoung Na, Cheolwon Lee, Hyun Kyu Kang, Heung Seok Jeon

**Affiliations:** 1 Department of Computer Engineering, Konkuk University, Chungju 27478, Korea; azammuminov92@gmail.com (A.M.); e10000won@gmail.com (C.L.); hkkang@kku.ac.kr (H.K.K.); 2 Global Leadership School, Handong Global University, Pohang 37554, Korea; soriru@handong.edu

**Keywords:** virtual fence, smart collar, livestock, machine learning, IoT, SVM

## Abstract

This paper describes our virtual fence system for goats. The present invention is a method of controlling goats without visible physical fences and monitoring their condition. Control occurs through affecting goats, using one or more sound signals and electric shocks when they attempt to enter a restricted zone. One of the best Machine Learning (ML) classifications named Support Vector Machines (SVM) is used to observe the condition. A virtual fence boundary can be of any geometrical shape. A smart collar on goats’ necks can be detected by using a virtual fence application. Each smart collar consists of a global positioning system (GPS), an XBee communication module, an mp3 player, and an electrical shocker. Stimuli and classification results are presented from on-farm experiments with a goat equipped with smart collar. Using the proposed stimuli methods, we showed that the probability of a goat receiving an electrical stimulus following an audio cue (dog and emergency sounds) was low (20%) and declined over the testing period. Besides, the RBF kernel-based SVM classification model classified lying behavior with an extremely high classification accuracy (*F-score* of 1), whilst grazing, running, walking, and standing behaviors were also classified with a high accuracy (*F-score* of 0.95, 0.97, 0.81, and 0.8, respectively).

## 1. Introduction

The Internet of Things (IoT) has the capability to transform the world we live in; more-efficient industries, connected cars, and smart cities are all components of the IoT equation. However, the application of technology like IoT in agriculture could have the most significant impact. Smart farming based on IoT technologies will enable growers and farmers to reduce waste and enhance productivity. So, what is smart farming? Smart farming is a capital-intensive and hi-tech system of growing agriculture cleanly and sustainably for the masses. It is the application of modern Communications Technology (ICT) to agriculture. In IoT-based smart farming, a system is built for monitoring the crop field and controlling animals with the help of sensors (light, humidity, temperature, soil moisture, etc.). The farmers can monitor the field conditions from anywhere. IoT-based smart farming is highly efficient when compared with the conventional approach [1,2].

RETRACTED

In some countries, the livestock industry has conducted various studies on smart farming using ICT. At first, Tiedemann and Quigley [3] began using a smart collar to control livestock in fragile environments. Their first work, published in 1990 [4], describes experiments in which cattle could be kept out of a region by remote manually applied audible and electrical stimulation. They note that cattle soon learn the association and keep out of the area, though sometimes cattle may go the wrong way. The cattle learn to associate the audible stimulus with the electrical one, and they speculate that the acoustic one may be sufficient after training. They did more comprehensive field-testing in 1992 with an improved smart collar. The idea of using GPS to automate the generation of stimuli was proposed by Marsh [5]. GPS technology is widely used for monitoring the position of wildlife. Anderson [6] built on the work of Marsh to include bilateral stimulation, consisting of different audible stimuli for each ear so that the animal can be better controlled. The actual stimulus applied appears to consist of audible tones followed by electric shocks. 

Behavior models classify the time series acquired from sensors by differentiating within the behavior classes based upon their unique motion characteristics. Models use sets of contiguous time series segments from either a three-axis accelerometer to represent the motion or orientation of the leg, neck, or head of the stocks; a microphone to capture the sound associated with animals’ behavior; or a GPS method to represent spatial movement patterns [7,8,9]. These models are generally known as time interval-based classifiers.

The simplest behavior models are known as binary models and detect a single behavioral incident [10,11,12,13] or differentiate between a set of behaviors. For instance, the eating behavior of cows was detected by counting relevant thresholds from the accelerometer data [12,13] or microphone data [10], whilst a moving average filter was used to separate the standing and walking behavior of cows [14]. Binary models are simple to develop given that they are comprised of few parameters, and, hence, easy to optimize. As models are developed to classify a higher number of behaviors, the class decision boundaries become increasingly complex. A high-dimensional parameter-space becomes necessary to discriminate between the classes. Consequently, machine learning methods are commonly adopted for problems with multiple behavior classes [7,9,10] given that they provide the necessary tools to estimate complex class decision boundaries in high-dimensional space.

RETRACTED

Virtual fencing technology has seen modern rapid approaches and has been demonstrated to be technically possible and near industrial availability for cattle (agersens.com). The algorithm that is used for cattle was initially developed by the Commonwealth Scientific and Industrial Research Organisation (CSIRO) Canberra, Australia. The virtual fencing devices use an algorithm that combines GPS with animal behavior to implement the virtual fence [15,16,17]. Similar to a physical fence, virtual fences assist in providing a boundary to contain animals, but unlike conventional fencing, they do not implement a physical barrier [18]. The potential for virtual fencing to alter the distribution of goat grazing has been demonstrated, but the perception and development of virtual fencing technology for goats is less advanced than for cattle. Research is required for virtual fence system development for goats, determining their activity, and improving the control of goats using sound stimuli with less electrical shockers. To fulfill the reminding goal, we have divided the virtual fence into three zones, such as safe, warning, and risk, and outside of the virtual fence we have called the escape area. The system uses different audio cues for each zone, except for the safe zone.

In this paper, we develop a virtual fence system for use in smart breeding. Our research is not limited to a virtual fence, and we have also added several new functions, such as observations of animals’ status using ML algorithms. Our IoT-based smart farming system is not only targeted at conventional, large farming operations, but it could also be employed for new levers to uplift other growing or common trends in agriculture, like organic farming and family farming, and enhance highly transparent farming. Unlike previous studies, we have provided the experiments in a large area to eliminate the potential use of a virtual fence as a spatial grazing technology for goats.

The remainder of this paper is organized as follows. Section 2 describes the summarized information about our virtual fence project. Section 3 extensively explains the implementation of the principal work of the smart collar side, a detailed construction of the smart collar hardware, and software tools. Moreover, it discusses the virtual fence application side and its objectives in our project and covers creating virtual fences, real-time communication with the smart collar, and real-time activity monitoring using SVM classification. Furthermore, an experiment schedule is clearly explained. Section 4 illustrates the experimental process and its result. Finally, Section 5 presents conclusions.

RETRACTED

## 2. The Virtual Fence Project

By creating a virtual fence project, we have tried to comprehend solutions for problems such as goat grazing or breeding over large paddocks. To make our project more helpful, we decided to include two main functions, such as monitoring and controlling goats.

### 2.1. Monitoring

Under the term of monitoring, there are two main features. The first one is monitoring the positions of the animals and the second is monitoring animals’ behavior. 

#### 2.1.1. Monitoring Animals Position

A variety of ways to obtain the animals’ position were observed in real-time, which helps to efficiently monitor animals in our application. Therefore, we chose the most common and popular GPS and geographic information systems (GIS) [19]. We have also included a GPS module in the smart collar (full information about smart collar hardware components written in Section 3).

The geographic information system is less well-known, but without GIS, GPS could not possibly be used to its full potential. GIS is a software program designed to store and manipulate the data that GPS accumulates [19].

#### 2.1.2. Monitoring Animals’ Behavior

Activity classification was added to track animals’ activity in real-time. One of the main reasons for adding activity classification is to create new functions, which gives additional information about the health status of the animal. To get a highly accurate classified result, we included the ML algorithm for our virtual fence system.

ML offers complementary data modeling techniques to those in classical statistics. In animal behavior, ML approaches can address otherwise intractable tasks, such as classifying species, individuals, vocalizations, or behaviors within complex data sets, which allows us to answer essential questions across animal behavior and their health status.

### 2.2. Controlling

Controlling animals is one of the most critical roles in our system. Controlling animals includes two main features: keeping animals inside a virtual fence and returning escaped animals to the virtual fence. If we can prevent escaping animals, returning escaped animals will not be a big problem.

#### Keeping Animals within Virtual Fences

First of all, to keep animals in an area, we need to create virtual fences. Our virtual fence is controllable through software; it is easy to install and move. A virtual fence is an arbitrary polygon drawn by the user, and it consists of an array of stiffness values of each vertex, as shown in Figure 1. The virtual fences are divided into three regions, as shown in Figure 1. Zone 1 is a safe area, Zone 2 is a warning area, and Zone 3 has been identified as a risk area, and outside of these areas we have called an escape area. Users can freely set up the distance between each area. In this study, the default value is set out considering the GPS error and the moving speed of the goat, in order for the distance between the safety and warning areas to be 5 m, and the distance between the warning and risk areas is 5 m as well. Control division of the virtual fence is designed to ensure the adequate control of goats on pastures. As was mentioned in the previous section, the stimulation of audio depends on the zone if the goat is in a safe area, free activity, and is not subject to any restrictions.

RETRACTED

To keep animals within virtual fences, the most common approaches, such as audio and electrical stimulus, were applied. However, our aim is to get a better result using conventional approaches. In view of this, different sounds and electrical stimuli were used with different straight in various areas.

## 3. Implementations

We have implemented a smart collar that is worn on the goats’ neck and a smart virtual fence application for users’ comfort to monitor and control their goats. The smart collar and virtual fence application communication is implemented as a centralized client-server architecture where the server component is responsible for the definition of the virtual fence zones with the decision algorithm.

### 3.1. The Virtual Fence Project: Smart Collar

The smart collar is composed of hardware and software solutions. We tried to make the most of cheaper and simpler devices; readily available components.

#### 3.1.1. The Smart Collar Hardware

Figure 2a shows the main components of a smart collar, and it consists of a speaker (3w), halters, and a main shield. Figure 2b presents the components of the central shield. These are Arduino NANO, a GPS module, an XBee communication module, MPU-6050 accelerometer and gyro sensors, mp3 player, and a high voltage igniter electrostatic generator (electrical shocker). A fully assembled collar on the goat neck is shown in Figure 3b. The following describes details about each module.

The Arduino Nano is a small, complete, and breadboard-friendly board based on the ATmega328. It has a pin layout that works well with the Mini or the Basic Stamp (TX, RX, ATN, and GND on one top, power, and ground on the other). The ATmega328 has a 32 kb memory (also with 2 kb used for the bootloader).

The Adafruit GPS unit is connected to the serial (TX1, RX0) port and 3v power port of the Arduino NANO. The Adafruit 66 Channel MTK3339 GPS Breakout Board V3 is built around the MTK3339 chipset, a no-nonsense, high-quality GPS module that can track up to 22 satellites on 66 channels, and has an excellent high-sensitivity receiver (−165 dB tracking) and built-in antenna. It can do up to 10 location updates a second for high speed, high sensitivity logging or tracking. Power usage is incredibly low, with a value of only 20 mA during navigation. 

RETRACTED

XBee Pro with the XBee USB Adapter Board is used to communicate with the server (virtual fence application), and the XBee USB Adapter is connected to digital pins (pin 8 and 9) and the 5v power port of Arduino NANO. This low-cost XBee USB Adapter Board comes in a partially assembled kit form and provides a cost-effective solution to interface a PC or microcontroller to any XBee module. The PC connection can be used to configure the XBee Module through Digi’s X-CTU software. The XBee Pro (higher-power) version of the popular XBee was used. This module is a series 1 (802.15.4 protocol) 60 mW wireless module, suitable for point-to-point, multipoint, and convertible to a mesh network point. This is much more powerful than the plain XBee modules with its feature of working for a long distance.

MPU-6050 is used to get smart collar accelerometer and gyro data. The MPU-6050 devices combine a three-axis gyroscope and a three-axis accelerometer on the same silicon die, together with an onboard Digital Motion Processor™ (DMP™), which processes complex six-axis MotionFusion algorithms. Additionally, it has an additional feature of an on-chip temperature sensor. It has an I2C bus interface to communicate with the microcontrollers, such as Arduino.

DFPlayer Mini (developed by the DFRobot Electronics in Shanghai, China) is used to play audio signals. The DFPlayer Mini module is a serial MP3 module that provides the perfect integrated MP3, WMV hardware decoding. Through simple serial commands, it specifies sound playing and other functions. The DFPlayer Mini is connected to digital pins (digital pin 2 and 3) and the 5v power port of Arduino NANO. Accordingly, we used an 8 GB memory card for DFPlayer to store mp3 files. 

The high voltage igniter electrostatic generator is used for electrical stimulus: the input voltage is dc 3–6 V, and the maximum output is 10 kv. The electrical shocker is connected to the digital pin 4 of the Arduino NANO through a small shocker controller circuit, which we created. A suitable high voltage wire with bulky insulation electrodes is installed on the left of the collar. Besides, two bold shape knobby metals are installed to deliver the electrical stimulus precisely to the skin (Figure 3a).

Future versions of the smart collar will most likely use the same modules as now, and will be used with a long-term battery and waterproof case to ensure the safety of the smart collar in any weather condition.

RETRACTED

#### 3.1.2. Software Infrastructure

The software process of the smart collar part is divided into two parts: sending and receiving data from the server. To satisfy communication, we use an XBee wireless network:

*(1) Sending data to the server:* The working process of the smart collar starts from reading XBee’s serial number. We decided to use the XBee serial number as the UUID of the device. The next step is reading data from sensors (such as GPS and accelerometer modules, including longitude, latitude, altitude, speed, accelerometer, and gyro) and sending it to the server. There are two kinds of outgoing messages. At first, the smart collar sends its first post as a request to the server for adding the animal to any virtual fence. When the server assigns a given animal to any field, the smart collar starts sending the second type of outgoing message. Each smart collar sends data at 1 Hz because the GPS satellites broadcast signals from space every second;

*(2) Handling incoming data:* After confirming the smart collar, the server checks the smart collar’s location and sends commands respectively. Incoming data from the server depends on the location of the goat. If the goat is inside the safety zone, the server sends the state number as zero; this means that sound coming out of the smart collar either stops or does not play. If the goat is in the warning zone, the server sends the appropriate commands to play sound. In the case of the animal being in the risk area or outside of the third fence, the server sends a command to use both electrical shocker and audio stimuli at the same time. The irritant sounds are stored in the DFPlayer memory card.

### 3.2. The Virtual Fence Project Server Side

We have developed a server that has an internet connection and an XBee communication module in order to eliminate the need for physical fences on farms, etc. The main tasks of our server are creating virtual fences using GPS coordinates on a remote computer, viewing and tracking the location of the goat through the wireless network in real time, and determining the animal deviated position in the intake area. These processes will be carefully examined in the coming sections.

#### 3.2.1. Virtual Fence

The server essentially defines fences as points on the surface of the earth. Thus, fences are infinite lines with a one-half plane defined as being desirable for animals. Virtual fences can be added or removed at any time, and several of them can be created at once from definitions stored in the database. Three fences can be combined to create convex polygonal shapes. When the GPS readings indicate that an animal has crossed the fence, a sound or electrical shock is triggered.

RETRACTED

#### 3.2.2. Virtual Fence Algorithms

The leading technologies that make a full virtual fence system are the distance measurement algorithm between the animal and the virtual fence, a Ray casting algorithm to check whether livestock exists in a region, and a Polygon Buffering algorithm used to divide the interval of a virtual fence.

Distance measurement algorithm: In general, the coordinate system used in GIS is not a rectangular coordinate system, but a spherical coordinate system. Google Maps in the virtual fence system uses the WGS84-based spherical Mercator projection method to project objects. Since the spherical Mercator projection deals with the earth as a sphere, the Euclidean distance formula used in Cartesian coordinates cannot be used. Generally, the distance between the two points $A\left(x_{1},y_{1}\right)$ and $B\left(x_{2},y_{2}\right)$ in the Euclidean space can be calculated by the following formula:

(1) $$\bar{AB}=\sqrt{{\left(x_{1}-x_{2}\right)}^{2}+{\left(y_{1}-y_{2}\right)}^{2}},$$

However, since the earth is round, the distance between two points projected on the map is a curved line on the surface. The Google Maps API provides a function that calculates the distance between two points in a spherical coordinate system using the Harversine algorithm [19]. Two points in the coordinate system of Google Maps are composed of latitude and longitude. 

The Ray Casting algorithm is used to check whether an animal is in the virtual fence area. The virtual fence is an arbitrary polygon, and the location of the livestock is an arbitrary coordinate value. This problem can be solved by the Point In Polygon (PIP) problem, which determines whether arbitrary coordinates are inside the polygon. A typical solution for PIP is the Ray Casting algorithm. The Ray Casting algorithm was proposed by Shimrat M. in 1962 [20], and it is also known as the Crossing Number algorithm or the Even-Odd Rule algorithm. The Ray Casting algorithm is mathematically proved through the Jordan Curve theory [21]. The Jordan Curve theory implies a single closed curve with the same connection with the circle.

#### 3.2.3. Physical Activity Classification

In the current study, goats’ activities are classified into five categories, as shown in Table 1. For a goat, ten time series acquired from the collar were analyzed including the three coordinates of the accelerometer and gyro, $x_{accx}\left(t\right),\;x_{accy}\left(t\right),\;x_{accz}\left(t\right)$, gyro, $x_{gyrox}\left(t\right),\;x_{gyroy}\left(t\right),\;x_{gyroz}\left(t\right),$ and the four-dimensional quaternion [22], $x_{quatx}\left(t\right),\;x_{quaty}\left(t\right),\;x_{quatz}\left(t\right),\;x_{quatw}\left(t\right)$ (they are x, y, z-axis and w-rotation amount). The I2Cdevlib Arduino library supports the four-dimensional quaternion calculation [23]; it plays the most important role in distinguishing between the five considered classes. In addition, the quaternion is used to monitor goats’ behavior in three-dimensional visualization.

RETRACTED

The ten time series were combined for classification:

(2) $$X\left(t\right)=\left[x_{accx}\left(t\right),\;x_{accy}\left(t\right),\;x_{accz}\left(t\right),x_{gyrox}\left(t\right),\;x_{gyroy}\left(t\right),\;x_{gyroz}\left(t\right),x_{quatx}\left(t\right),\;x_{quaty}\left(t\right),\;x_{quatz}\left(t\right),\;x_{quatw}\left(t\right)\right]$$

where X(t) is an array of the ten time series at a particular time sample index t.

The ML algorithm named Support Vector Machines was used to classify a goat’s activity. We used SVM because it copes well with small and unbalanced data. SVM is a classifier that has been frequently used in machine learning and pattern recognition and is hence a linear classifier in the use of hyperplane with the maximum margin as the decision boundary [24,25]. The linear classification SVM model is shown in Equation (3).

(3) $$d\left(w,\;x,\;b\right)=\langle w\cdot x\rangle +b=\overset{S}{\underset{i=1}{\sum }}w_{i}\cdot x_{i}+b$$

Here, S is the number of the Support Vector, x is a feature vector representing sample data, and w and b are parameter values that determine the hyperplane. The linear classifier tends to show a high performance if a feature vector is categorized as linear.

However, our data for classification is high-dimensional. It can be classified better with non-linear classification techniques. In this case, the Kernel Trick technique was used to classify high-dimensional data. Four types of Kernel function in SVM are represented in Table 2. The most common one is the Radial Basis Function (RBF) kernel [24]. So, in this paper, we used the RBF kernel to classify goats’ activities.

We have developed two different features using SVM. The first one makes a predictive model and checks the prediction accuracy, as illustrated in Figure 4a [26]. The second one performs the real-time classification, as shown in Figure 4b [26].

#### 3.2.4. Stimulus and Stimuli Methods

We realized some options for sound stimulus, such as “static volume”, “dynamic volume”, and “dynamic sound”, as shown in Figure 5. The smart collars are capable of administering different sounds with different volumes in dB (76–108 dB, 2.9 kHz) for each zone, as warning, risk, and escape zones. Moreover, we determined a different approach for a pulsing electrical stimulus to the goat—the electrical stimulus strength changes, depending on the distance from zones. The system uses the shocker in emergency situations, i.e., when it is complicated returning animals to the safety zone by applying a single audio cue because using an electrical shocker in goats several times may negatively affect their health and body. The shocker mode straight changes from 0V to 10 kV. In our situation, the shocker mode changes by the distance inside of the risk area from 4 kV to 10 kV (it pulses during 200 ms per second), and it uses maximum power outside of a virtual fence (escape zone). The sounds for each zone used in our experiments are included in Table 3.

RETRACTED

Five different audio cues sets are used (Table 3). The sounds in the first column are only used only in the warning zone, as well as other column sounds. All three dog sounds are taken from different individuals with different scarring attributes, and other sound sets are the same. This helps escape from the adaptation behavior of goats for sounds. We called siren, buzzer, etc. sounds the “Emergency Signal” and the “Ultrasounds” are the thin unpleasant sounds.

#### 3.2.5. Server GUI (Graphical User Interface)

Most of the advantages of our project are more accessible to establish available server settings and control smart collars. When a user starts the server for the first time, the server configuration will be presented as a default (static). On the other hand, there are dynamic settings; these allow users to configure the server according to their desires (Figure 5). Furthermore, we have developed 3D monitoring of a goat position using four-dimensional quaternion data; this gives a great chance to observe goats’ poses in real-time, as shown in Figure 6. Figure 7 shows a GUI that includes one animal, which is outside of the area.

## 4. Physical Experimental Results

Unlike earlier studies, our temporarily drawn virtual fence for the experiment is not limited by the sides (as presented in Figure 7), and the experimental goats may move in any directions they want. 

Goats have leadership behavior in a domestic goat group that modifies the activity of the group. Usually, the adult female occupies leadership positions [27], which is also seen in sheep [28].

For the physical experiment, ten goats were chosen, and we installed the smart collar on the leader goat of the herd. The reason for choosing ten goats is that goats are always used to being with a herd of goats. It might have affected the experiment result if we chose one.

### 4.1. Experimental Environments

Firstly, we chose a place on an Uzbekistan (Shirin, Sirdaryo, Uzbekistan) farm to conduct physical experiments located at 40°14′36.2″ N 69°05′40.5″ E. We prefer to choose farms with grasses and large areas, as shown in Figure 8, which gives the best chance to observe significant experimental results. In all field experiments, we visually observed the behavior of individual goats with the smart collar (as illustrated in Figure 3b) and several experiments were conducted on some days. However, for the current study, we have conducted the experiment in seven days from 8 a.m. to 6 p.m. Five days were spent on the stimulation experiment, and on the remaining two days, we collected the necessary data for the behavior classification. All the experimental processes were observed and recorded with a video camera.

RETRACTED

### 4.2. Stimulation Experiment

In the current research, we tried to control goats using several types of sounds to ensure less usage of the electrical stimulus. The sounds used in our experiments are shown in Table 3.

Mainly five different experiments have been carried out using five different stimuli. As the goat entered the warning zone, a 1 s audio cue was delivered. If the goat displayed either of the following responses: stopping, turning away, or backing up, the audio cue was ceased before 2 s elapsed. If the goat failed to respond to the audio cue (running forward or entering the next (risk) zone) after 2 s, then an immediate audio cue and electrical stimulus (with strength from 4 kv to 10 kV depending on the distance from warning zone line. It pulses during 200 ms per second) were applied for 1 s. If the animal ran towards the escape zone, the audio cues and stimulus were not reapplied until the animal had calmed down, i.e., stopped running. Once the animal was calm, if they proceeded further into the escape zone, the audio cue and electrical stimulus (with maximum strength) were reapplied until they turned and exited the exclusion zone.

During the five days, the smart collar installed goat had a higher percentage of audio cues than electrical stimuli. Within each day, each audio cue showed a different effectiveness. Table 4 illustrates that the usage percentage of dog and emergency sounds is higher than other audio cues. The behavior response for each stimulus is presented in Table 5 and Table 6.

### 4.3. SVM Classification Experiment

#### 4.3.1. Collecting Data for Goat Behavior

The smart collar was programmed to send data at 1 Hz (i.e., 86,400 data points/day). On the last two days of the experiment, we decided to collect data for SVM classification without any stimuli. Five behaviors, such as standing, walking, running, grazing, and lying, were recorded during the experiment (Table 1). The smart collar recorded the data every 1 s between the hours of 8 a.m. and 6 p.m.

RETRACTED

#### 4.3.2. SVM Classification Results

RBF kernel SVM needs *gamma* and *C* parameters [29]. In our experiments, we used the SVM grid search function of the scikit-learn library in Python [30]. The function finds the effective parameters of the *gamma* and *C* of the RBF kernel SVM. The best parameters defined from the function are ${\{}^{\prime }C^{\prime }:1.0,{}^{\prime }gamma^{\prime }:1.0\}$ with a score 0.91. The parameter selecting process is shown in Figure 9. The first plot is a visualization of the decision function for a variety of parameter values on a simplified classification problem involving only two input features and two possible target classes (binary classification). It is not possible to create this kind of plot for problems with more features or target classes. The second plot is a heatmap of the classifier’s cross-validation accuracy as a function of *C* and *gamma*. We explored a relatively large grid for illustration purposes. In practice, a logarithmic grid from $10^{-3}$ to $10^{3}$ is usually sufficient. If the best parameters lie on the boundaries of the grid, it can be extended in that direction in a subsequent search.

After obtaining some goat activity data from the last experiment, we made training sets for SVM. The training sets consist of 2000 data points for each condition, so the total training set data is 10,000. To evaluate the accuracy of SVM, 200 test datasets are used for each condition, and the total data is 1000. The result of total accuracy is 91% (the results are presented in Table 7). The performance was evaluated using the *F*-score metric, recall (*R*), and precision (*P*) [31]:

(4) $$F=\frac{2*P*R}{P+R}$$

(5) $$R=\frac{truepos}{truepos+falseneg}$$

(6) $$P=\frac{truepos}{truepos+falsepos}$$

where *truepos* was the number of intervals from the class that was correctly classified, *falsepos* was the number of intervals from another class that was incorrectly classified as the class, and *falseneg* was the number of intervals belonging to the class that was classified as another class. The recall is the fraction of time intervals belonging to a class that was correctly classified, and precision is the fraction of intervals from a classification that was correct. The *F*-score statistic was the harmonic mean of the precision and recall ranging between 0 and 1. The final *F*-score of the classifier was computed by averaging the individual *F*-scores of the five folds.

## 5. Conclusions

In this paper, we introduced the concept of a virtual fence, such as a server and smart collar, which applies a stimulus to an animal as a function of its pose concerning one or more fence lines. The fence algorithm is implemented by a small position-aware computer device worn by the animal, which we refer to as a smart collar. We described a simulator based on potential fields and stateful animal models whose parameters are informed by field observations and track data obtained from the smart collar. We considered the effect of sound and electric shocker stimuli on the goat, but have had questions due to habituation. Moreover, we considered the option of infrequently using an electric shock stimulus because we thought it would be fierce if we use it often. Instead, we have divided the virtual fence into three zones as a safe area, warning area, and risk area and different audio cues have been used to scare and control goats. Users can select the sound set from the list manually in order to avoid the habituation of goats to the same sounds. The goat in this study had a low probability (20%) of receiving an electrical stimulus, even before learning to associate the audio cue with the electrical stimulus. Following the removal of the virtual fence on the last two days, animals were quick to cross the location to access the other part of the experimental area, indicating that the animals studied responded to the cues rather than the location of the virtual fence. In this study, a leader goat was given an audible warning before the utilization of an electrical stimulus, which was only applied if the goat did not turn or stop on the warning zone on the audio. The goat had a large number of interactions with the fence and was willing to spend time close to the virtual fence location, but was still successfully restricted to a portion of the paddock.

RETRACTED

The classification performance for five of the goat behavior classes; grazing, walking, running, standing, and lying, were presented in this analysis. The RBF kernel-based SVM classification offered a significantly high classification performance for the five goat behaviors, as shown in Table 5. For three of the behavior classes; grazing, running, and lying, the classification achieved a greater F-score performance than the other two classes.

However, the study by Markus et al. [32], who compared a conventional electric fence with a virtual fence while restricting access of cattle to the trough, found that cattle trained on a virtual fence did not want to cross their location after removal. This study showed that cattle were wary of the place where the virtual fence was installed and that the virtual fence may affect the behavior of livestock, even after its removal. The study by Markus et al. [32] exclusively implemented an electrical stimulus without sound; cattle only had visual and spatial stimuli to associate with the virtual fence. Therefore, it is clear why the cattle would not like to cross a location that is associated with a negative stimulus since the only sign that they are going to receive a negative incentive is from the position itself. In our study, this reaction was not observed. Longer-term studies need to be conducted to discover the effect of virtual fencing on typical patterns of animal behavior.

Our future work has many different directions and different locations. We wish to create new functions which give more information about the health of animals using developed SVM classification. Furthermore, we are going to implement a new feature, which includes moving goats from one area to another using temporary virtual fences. These models will lead to a better understanding of animal behavior and control at the individual and group level, which has the potential to impact not only the goat industry, but more broadly, agriculture.

## Figures and Tables

**Figure 1:** Virtual Fence.

**Figure 2:** Virtual Fence Smart Collar: (**a**) The main components of a collar, consisting of a speaker (3w), battery, electrical shocker, halters, and main shield; (**b**) the components of the smart collar are an Arduino NANO, XBee communication module, electrical shocker controller, GPS module, accelerometer sensor, SD card reader, and mp3 player with 8 GB memory card.

**Figure 3:** (**a**) Electrical shocker electrodes position of the smart collar. (**b**) Fully assembled smart collar worn on the goat.

**Figure 4:** A typical supervised learning workflow. (**a**) Exploratory data analysis is followed by a feature extraction step to derive putative discriminatory variables. The observations are split into training and testing data sets, and the predictive model trains on the training data set. Training involves the SVM model generalization step. Finally, the model’s generalization performance computes using the testing dataset. (**b**) Real-time classification workflow. SVM real-time classification using a predictive model.

**Figure 5:** Virtual Fence settings GUI.

**Figure 6:** 3D Monitoring of a goat illustrated as a cube (in the top left corner of the picture). A real-time graph of all incoming data from the smart collar. It is possible to see historical data by applying the period of date and time.

**Figure 7:** Virtual Fence GUI with an animal outside of the virtual fence.

**Figure 8:** Experimental area with a size of 96117 m^2^.

**Figure 9:** RBF kernel SVM *gamma* and *C* parameters selection process. (**a**) Visualization of the decision function for a variety of parameter values. (**b**) A heatmap of the classifier’s cross-validation accuracy as a function of *C* and *gamma*.

RETRACTED

**Table 1:** Activity classes of goat. The five defined in this study; standing, walking, running, grazing, and lying, were described.

Class	Description
Standing	A goat is normally standing
Walking	A moving goat that is taking steps with the head in an upright position
Running	A faster-moving goat with the frequent body shake
Grazing	The head of the goat is tilted downwards and positioned near the ground. The goat is either taking bites of the pasture or searching for the pasture
Lying	A goat that is lying

**Table 2:** SVM Kernel Formulas.

Kernel	$K\left(x_{i},\;x_{j}\right)$
Linear	$X_{i}^{T},\;X_{j}$
Polynominal	${\left(\gamma X_{i}^{T}X_{j}+r\right)}^{d},\gamma >0$
Radial Basis Function (RBF)	exp$\left(-\gamma \|X_{i}-X_{j}\|{}^{2}\right),\gamma >0$
Sigmoid	$\tanh\left(\gamma X_{i}^{T}X_{j}+r\right)$

**Table 3:** List of sound stimuli.

Warning Zone	Risk Zone	Escape Zone
Dog-1	Dog-2	Dog-3
Lion-1	Lion-2	Lion-3
Tiger-1	Tiger-2	Tiger-3
Emergency Signal-1	Emergency Signal-2	Emergency Signal-3
Ultrasound-1	Ultrasound-2	Ultrasound-3

**Table 4:** Contingency table of the number of times the electrical stimulus was or was not applied to the goat, following an audio cue during the stimuli tests.

Experiment Day	Audio Type		Sound	Electrical Stimulus
1	Dog sound	Count	53	14
		Percentage	79.10%	20.90%
2	Lion sound	Count	27	42
		Percentage	39.13%	60.87%
3	Tiger sound	Count	23	40
		Percentage	36.51%	63.49%
4	Emergency sound	Count	49	12
		Percentage	80.33%	19.67%
5	Ultrasound	Count	18	41
		Percentage	30.51%	69.49%

**Table 5:** Count of behaviors from a goat, presented in response to the audio cues over the five days the virtual fence was experimented.

Response to Audio	1st Day	2nd Day	3rd Day	4th Day	5th Day
Continue forward	1	23	18	2	15
Turn	6	0	0	5	0
Stop	10	1	2	8	2
Grazing	36	2	3	33	1
Flinch	0	1	0	1	0
Total interactions	53	27	23	49	18

**Table 6:** Contingency table of the number of times the electrical stimulus was or was not applied to the goat, following an audio cue during the stimuli tests.

Response to Electrical Stimulus	1st Day	2nd Day	3rd Day	4th Day	5th Day
Turn	2	10	9	3	10
Jump	8	21	19	5	17
Stop	2	3	2	3	5
Flinch	2	5	4	1	6
No reaction	0	3	6	0	3
Total interactions	14	42	40	12	41

**Table 7:** Accuracy of the SVM classification.

Evaluation Report	Standing	Walking	Running	Grazing	Lying	Total Accuracy
Precision	0.93	0.75	1	0.9	1	0.92
Recall	0.7	0.9	0.95	1	1	0.91
F-score	0.8	0.81	0.97	0.95	1	0.91
Data size	200	200	200	200	200	1000
